The article "Clinical Study of Heart Failure with Left Ventricular Ejection Fraction Regimen Treated with Entresto" was retracted in 2023. Reasons: signs of a paper mill; suspected computer-generated content; unreliable results or conclusions; concerns about the data.

# Clinical Study of Heart Failure with Left Ventricular Ejection Fraction Regimen Treated with Entresto

**DOI:** 10.1155/2022/4164089

**Published:** 2022-08-09

**Authors:** Mingjun Feng, Bin He, Binhao Wang, Xiaomin Chen, Huimin Chu

**Affiliations:** ^1^Arrhythmia Center, Ningbo First Hospital, Ningbo 315000, China; ^2^Key Laboratory of Precision Medicine for Atherosclerotic Diseases of Zhejiang Province, China

## Abstract

Heart failure is a group of syndromes caused by various cardiac structural or functional disorders leading to impaired ventricular filling and (or) ejection capacity. Because of decreased ventricular systolic function and impaired ejection function, the amount of cardiac output cannot meet the body's metabolic needs; organ and tissue blood perfusion is insufficient; at the same time, pulmonary circulation and (or) systemic circulation congestion; the clinical manifestations are mainly dyspnea and weakness but restricted physical activity and edema. Treatment of the disease should include preventing and delaying the onset of wails, relieving symptoms of clinical wails, improving its long-term prognosis, and reducing mortality. The aim of the study is to observe the efficacy and safety of Entresto in the treatment of left ventricular ejection fraction heart failure (HFpEF). Seventy-eight patients with HFpEF treated in our hospital from October 2017 to April 2018 were randomized into a treatment group (Entresto 50 mg + basic treatment, *n* = 39) and a control group (basic treatment, *n* = 39). The course of treatment was ten weeks. The levels of brain natriuretic peptide (BNP) and echocardiographic indicators (LVMI, LVEF, LVEDD, LVESD, E/E′ Ratio, E/A ratio, DT), 6-minute walking test (6MWD), and Minnesota Quality of Life Scale (MLHFQ) were analyzed before and after treatment. LVMI, LVEF, LVEDD, LVESD, E/E′ ratio, E/A ratio, DT, and BNP were all significantly improved in the Entresto group after treatment. In the control group, except for LVEDD, LVESD, the E/A ratio, and BNP, other indicators were significantly improved after treatment (*P* < 0.05). Posttreatment, both groups had significantly improved 6MWD and MLHFQ scores (*P* < 0.05). Differences in these parameters between the two groups were statistically significant (*P* < 0.05). After treatment, the levels of NE, AngII, ALD, and MMP-9 in the two groups were decreased (*P* < 0.05), with the lower lever in the treatment group (*P* < 0.05). The effective rate was 76.92% in the control group and 94.87% in the Entresto group, and this rate difference was statistically significant (*P* < 0.05). The number of patients re-hospitalized due to cardiovascular events was 2 (the Entresto group) vs. 7 (the control group) cases; worsening of heart failure was observed in 1 patient (the Entresto group) vs. 6 (the control group), and the difference between the two groups was statistically significant (*P* < 0.05). However, the incidence of adverse reactions between the two groups was not statistically significant. Entresto can significantly improve left ventricular diastolic function in heart failure patients with preserved left ventricular ejection fraction and improve quality of life. This treatment is safe and effective and worthy of clinical application. This trail is registered with ChiCTR2000031486. This trial was approved by the Chinese Clinical Trial Registry (clinical trial number: ChiCTR2000031486). The registration number of this study is 2022-R008.

The article "Clinical Study of Heart Failure with Left Ventricular Ejection Fraction Regimen Treated with Entresto" was retracted in 2023. Reasons: signs of a paper mill; suspected computer-generated content; unreliable results or conclusions; concerns about the data.

## 1. Introduction

Heart failure (HF) is a group of clinical syndromes in which ventricular filling or ejection disorders with various leads to metabolic and circulatory disorders in tissues and organs throughout the body. Such outcomes are the fate of all patients with heart disease [1]. Heart failure with preserved left ventricular ejection fraction (HFpEF) is also called left ventricular diastolic heart failure. It has long been widely believed that heart failure is caused by left ventricular systolic dysfunction. With the deepening of research, clinical evidence indicates that some patients with heart failure can still maintain a relatively normal ejection fraction. Heart failure with preserved left ventricular ejection fraction (HF PEF) refers to heart failure with normal or near normal LVEF (>0.5 or 0.45) but with signs or symptoms and is often referred to as diastolic heart failure, the specific pathophysiological mechanism of which is currently ill-defined and is generally believed to be due to impaired left ventricular diastolic active relaxation capacity and reduced myocardial compliance, causes impaired diastolic filling of the left ventricle and a reduction in stroke volume, leading to heart failure in the setting of increased left ventricular end-diastolic pressure. The population incidence of HFPEF is higher than previously recognized and the prognosis is worse than envisioned, and it should be given high priority.

Risk factors for developing heart failure are primary cardiac disease, diabetes mellitus, atherosclerotic disease, and having any factor that can aggravate the disease will aggravate or induce the development of heart failure. (1) Primary disorders of the heart. In the clinic, there are common diseases such as coronary heart disease, hypertension, and myocardial ischemia, which will cause heart failure. Meanwhile, hypertensive people are at a higher risk of developing heart failure than nonhypertensive people, and the higher the level of blood pressure, the older the age and the longer the duration of hypertension, the higher the incidence of heart failure. (2) Diabetes. The development of diabetes increases the odds of heart failure and it affects the prognosis of heart failure. (3) Atherosclerotic disease. Heart failure is more likely to occur when patients present with atherosclerotic disease of the coronary, cerebral, and peripheral vessels. (4) Common triggers include excessive physical effort, agitation, excessive sodium salt intake, arrhythmias, pregnancy or childbirth, too rapid infusion or transfusion of fluids, too much, taking certain medications, and when an infection, particularly a respiratory infection, can create an increased burden on the heart, which can trigger the development of heart failure.

The article "Clinical Study of Heart Failure with Left Ventricular Ejection Fraction Regimen Treated with Entresto" was retracted in 2023. Reasons: signs of a paper mill; suspected computer-generated content; unreliable results or conclusions; concerns about the data.

As a result, heart failure caused by diastolic dysfunction has become a research hotspot [2]. Epidemiological surveys show that there are about 13 million heart failure patients in China, of which HFpEF accounts for about 56%, and it is increasing year by year. Older women are a high-risk population [3]. In recent years, clinical trial results using drugs to reduce heart failure mortality have not been satisfactory [4, 5], so there is an urgent need for a safe and effective therapy for the treatment of HFpEF. Entresto is an angiotensin receptor-neprilysin inhibitor (ARNIs), a compound preparation composed of sacubitril and valsartan at a ratio of 1 : 1. It acts by relaxing blood vessels and preventing and reversing cardiovascular remodeling. After many clinical trials, the U.S. “2016 Heart Failure New Drug Therapy Guidelines” listed Entresto as a Class I recommendation for the treatment of heart failure. This study adopted a prospective randomized controlled trial design to observe the efficacy and safety of Entresto in the treatment of HFpEF.

## 2. Materials and Methods

### 2.1. General Information

Patients with HFpEF admitted to the Department of Cardiology of our hospital from October 2017 to April 2018 were selected as the research objects. The inclusion criteria were as follows: (1) age 40 to 75 years; (2) meet the diagnostic criteria for HFpEF; (3) conscious, volunteer to participate, and able to cooperate well with the trial; (4) NYHA cardiac function classification is II∼III; and (5) left ventricular ejection fraction (LVEF) 40–50%, left ventricular end-diastolic volume index (LVEDVI) < 97 ml/m^2^. The exclusion criteria were as follows: (1) left ventricular ejection fraction (LVEF) < 40%; (2) heart failure caused by liver and kidney failure; (3) history of allergy to sacubitril or valsartan; (4) right ventricular failure caused by chronic obstructive pulmonary disease, pericardial disease or other reasons; (5) patients with malignant tumors, hematological diseases and autoimmune diseases; and (6) pregnant or lactating women. A total of 78 patients meeting the criteria were enrolled, including 31 male and 47 female, aged 42–75 years old, with an average age of (60.52 ± 8.65 years). The patients were randomly divided into control and treatment groups (*n* = 39 each). Gender, body mass index, blood pressure, and NYHA classification were all matched. Our hospital's ethics committee approved this study, and all selected participants voluntarily signed an informed consent form. The registration number of this study is 2022-R008.

The article "Clinical Study of Heart Failure with Left Ventricular Ejection Fraction Regimen Treated with Entresto" was retracted in 2023. Reasons: signs of a paper mill; suspected computer-generated content; unreliable results or conclusions; concerns about the data.

### 2.2. Diagnostic Criteria

According to the 2014 “Chinese Heart Failure diagnosis and Treatment Guidelines” [6], combined with the 2013 version of the “ACCF/AHA Heart Failure Management Guidelines” [7], the following diagnoses are met: (1) have typical symptoms or signs of heart failure, meeting Framingham's diagnostic criteria for heart failure. 1 Nocturnal paroxysmal dyspnea and/or waking up from sleep; 2. increased jugular vein irritability or pulsation; 3. diminished rales and/or respiratory sounds in the lungs, especially in the bilateral lung bases; 4. cardiac enlargement on imaging; 5. acute pulmonary edema; 6. third heart sound gallop; 7. elevated jugular venous pressure >16 cmH2O; 8. positive hepatojugular reflux sign; and 9. weight loss > 4.5 kg within 5 days of treatment. Chronic congestive heart failure (CHF) was diagnosed when 2 conditions were met). (2) The left ventricle size is normal, the systolic function is normal or slightly abnormal, and the LVEF is 40–50%. (3) BNP > 200 pg/ml. (4) Echocardiograms suggest diastolic dysfunction, E/E′ ≥ 8. NYHA Heart Function Classification: Grade I : Unrestricted activities, as regular physical activity will not cause shortness of breath, palpitations, or fatigue. Grade II : Slightly restricted activities, relieved during rest, daily activities can cause shortness of breath, heart palpitations, or fatigue. Grade III : Restricted activities, no symptoms at rest, and a small amount of activity can cause significant shortness of breath, palpitations, or fatigue. Grade IV : Symptoms are evident during rest and aggravated during activity.

### 2.3. Treatment

The two groups of patients were evaluated after enrollment and received general treatments such as oxygen inhalation and rest. Conventional antiheart failure drugs were treated for more than two weeks. The control group received basic pharmacological treatments including Diovan, *β*-blockers, CCB, nitrate drugs, antiplatelet drugs, etc. In the treatment group, 50 mg sacubitril and valsartan sodium tablets were added to *β*-blockers, CCB, nitrate drugs, and antiplatelet drugs (Entresto: 50 mg/tablet, manufacturer: Novartis Pharma Stein AG) orally, twice a day. All patients were evaluated after ten weeks of treatment. These are two drugs with different mechanisms of action and the efficacy after the combination is superior to either alone and does not occur.

The article "Clinical Study of Heart Failure with Left Ventricular Ejection Fraction Regimen Treated with Entresto" was retracted in 2023. Reasons: signs of a paper mill; suspected computer-generated content; unreliable results or conclusions; concerns about the data.

### 2.4. Observation Index

The observation indexes were as follows:

1. Echocardiography before and after treatment, inspection indicators were left ventricular mass index (LVMI), left ventricular ejection fraction (LVEF), left ventricular end-systolic diameter (LVESD), left ventricular end-diastolic diameter (LVEDD), E/E′ Ratio, E/A ratio, E peak deceleration time (DT).
2. Laboratory test indicators: plasma brain natriuretic peptide (BNP) levels, blood lipids TC, TG, HDL-C, LDL-C levels. Serum levels of neutrophil elastase (NE), angiotensin II (AngII), aldosterone (ALD), and matrix metalloproteinase 9 (MMP-9).
3. Clinical evaluation: The 6-minute walk test (6MWD) was used to evaluate the patient's heart function before and after treatment.
4. Quality of life assessment: The Minnesota Living with Heart Failure Questionnaire (MLHFQ) was used to assess the quality of life before and after treatment.
5. Composite clinical endpoints: incidence of worsening heart failure, myocardial infarction, cardiovascular rehospitalization, cardiovascular death, etc.

### 2.5. Efficacy Evaluation Criteria

To evaluate treatment efficacy, we referred to the Heart Function Evaluation Standard established by the European Heart Association in 2007. To be deemed “Significantly effective,” the improvement of cardiac function must be greater than or equal to Grade 2; “Effective” is defined by an improvement of cardiac function greater than Grade 1 and less than Grade 2. An “invalid” evaluation reflects no improvement in cardiac function. Effective rate = (markedly effective + effective)/total number of patients × 100%.

### 2.6. Statistical Analysis

The statistical software SPSS 19.0 was used to statistically analyze obtained data. The count data were compared using a chi-square test, a rank sum test compared the rank data, and the measurement data were compared using a *t*-test. *P* < 0.05 was considered statistically significant.

## 3. Results

### 3.1. Comparison of Echocardiographic Indexes of the Two Groups of Patients before and after Treatment

The results showed that there was no statistically significant difference in LVMI, LVEF, LVEDD, LVESD, E/E′ ratio, E/A ratio, or DT between the two groups before treatment (*P* > 0.05); the LVEF, LVEDD, LVESD, E/E′ ratio, E/A ratio, and DT of the Entresto group were significantly improved after treatment (*P* < 0.05); there was no significant difference in LVEDD, LVESD, and E/A ratio in the control group between pre- and posttreatment (*P* > 0.05). There were significant differences in all the abovementioned parameters posttreatment between the two groups (*P* < 0.05), indicating that the two treatment options can improve the left ventricular ejection fraction and left ventricular diastolic function of patients with HFpEF; however, the outcome of the Entresto group is better than that of the control group as shown in Table 1.

The article "Clinical Study of Heart Failure with Left Ventricular Ejection Fraction Regimen Treated with Entresto" was retracted in 2023. Reasons: signs of a paper mill; suspected computer-generated content; unreliable results or conclusions; concerns about the data.

### 3.2. Comparison of Plasma BNP Levels between the Two Groups of Patients before and after Treatment

There was no significant difference in plasma BNP levels between the two groups before treatment (*P* > 0.05). Following treatment, BNP was significantly improved compared to before treatment (*P* < 0.05), and the difference in the control group was not significant (*P* > 0.05). However, compared with each other after treatment, the difference was statistically significant (*P* < 0.05) as shown in Table 2.

### 3.3. Comparison of the 6-Minute Walk Distance (6MWD) and Quality of Life between the Two Groups before and after Treatment

Before treatment, 6MWD and MLHFQ scores were not significantly different between the two groups (*P* > 0.05). After treatment, both groups were significantly improved compared to before treatment (*P* < 0.05). The difference between the groups was statistically significant (*P* < 0.05) as shown in Table 3.

### 3.4. Comparison of Serum Factor Levels between the Two Groups before and after Treatment

There was no significant difference in the levels of NE, AngII, ALD, and MMP-9 between the two groups before treatment (*P* > 0.05). After treatment, the levels of these factors in both groups were decreased (*P* < 0.05), with the lower level in the treatment group (*P* < 0.05), as shown in Table 4.

### 3.5. Comparison of the Curative Effect on the Cardiac Function between Two Groups

The effective rate of the control group was 76.92%, and the treatment group was 94.87%. The difference between the two groups was statistically significant (*P* < 0.05) as shown in Table 5.

### 3.6. Comparison of Composite Clinical Endpoints between the Two Groups of Patients

In the Entresto group/control group, there were 2/7 cases re-hospitalized due to cardiovascular events, and 1/6 patients experienced worsening heart failure. The difference between the two groups was statistically significant (*P* < 0.05). There was no statistically significant difference in the incidence of adverse reactions between the two groups (*P* > 0.05) as shown in Table 6. In terms of safety, the most common adverse reaction was dizziness, with 1 case in the Entresto group and 3 cases in the control group. One case in each of the two groups exhibited impairment of kidney function. One case with hyperkalemia was identified in the Entresto group. There was one case diagnosed with hypotension in each group.

The article "Clinical Study of Heart Failure with Left Ventricular Ejection Fraction Regimen Treated with Entresto" was retracted in 2023. Reasons: signs of a paper mill; suspected computer-generated content; unreliable results or conclusions; concerns about the data.

## 4. Discussion

Heart failure is not an independent disease but the final stage of developing all organic heart diseases. Nevertheless, it was found that some patients with heart failure could still maintain a relatively normal ejection fraction. The European Society of Cardiology “Guidelines for the diagnosis and treatment of acute and chronic heart failure 2008” recommends that this type of heart failure is called HFpEF. Studies have shown that the left ventricular end-diastolic pressure in patients with HFpEF increases, causing pulmonary or systemic venous congestion, and increased susceptibility to nighttime paroxysmal dyspnea, cough, fatigue, etc., which negatively affects their quality of life and threatens their health and survival [8]. Gender, old age, left ventricular hypertrophy, and hypertension are recognized risk factors for HFpEF [9].

The pathogenesis of HFpEF remains unclear and left ventricular diastolic dysfunction cannot fully explain the symptoms of dyspnea and systolic heart failure in clinical patients [10]. Experimental studies found that arterial stiffness in HFpEF patients was significantly increased, ventricular diastolic function was impaired, and arterial compliance decreased. This sequela leads to increased cardiac ejection resistance, left ventricular filling disorder during diastole, elevated left ventricular end-diastolic pressure, reduced stroke volume, and the risk of heart failure significantly increases [11]. Therefore, most researchers believe that ventricular diastolic dysfunction, decreased arterial compliance, and increased stiffness may be some of the causes of HFpEF [10, 12, 13]. At present, there are no effective treatments or drugs that can effectively improve early diastolic heart failure in clinical practice. Conventional drug treatments are not satisfactory, and the prognosis is poor [14]. The treatment of HFpEF has become a worldwide clinical challenge [15].

Entresto is the world's first angiotensin receptor- neprilysin inhibitors (ARNIs) developed by Novartis. It is mainly composed of valsartan and sacubitril combined in a sodium salt complex at a ratio of 1 : 1 [16, 17]. Among them, sacubitril is a prodrug of an enkephalinase (NEP) inhibitor. The drug can reduce the pre- and post-load of the heart, improve ventricular remodeling, and prevent heart failure by antagonizing AT1, inhibiting angiotensin II receptors and enkephalinase. In a multicenter randomized, parallel, and controlled phase II clinical trial involving a total of 301 patients with heart failure with reduced left ventricular ejection fraction, left atrial volume, and diameter of the Entresto group after 36 weeks of treatment was significantly smaller than the control group [18]. A more extensive phase III clinical trial enrolled 8442 patients with heart failure with reduced left ventricular ejection fraction. Enalapril was used as a control and patients were treated for 4 weeks. The results showed that Entresto reduced clinical endpoint events and improved clinical outcomes. Symptoms and activity endurance were also significantly better posttreatment with Entresto than with enalapril [19]. The 2016 European Society of Cardiology (ESC) guidelines for the diagnosis and treatment of acute and chronic heart failure and the 2017 ACC/AHA/HFSA Guideline for Management of Heart Failure Update listed Entresto as a Class I recommendation for the treatment of HFREF. Nioxin also demonstrated unparalleled superiority in the treatment of HFpEF patients. The PARAMOUNT study published in 2012 [20] and its subsequent analysis showed [21] that patients with heart failure (HFpEF) showed preserved ejection fraction after 36 weeks of follow-up. The levels of NT-proBNP and high-sensitivity troponin T (hs-TnT) were also significantly reduced after the treatment by Entresto. In addition, the incidence of serious adverse events in the Entresto group was lower than that of valsartan (15% vs. 20%). However, the small-sample PARAMOUNT study did not use the clinical benefit as the endpoint but only used laboratory indicators as a surrogate endpoint. Therefore, whether Entresto can ultimately improve clinical outcomes in patients with HFpEF requires further study with larger samples.

The article "Clinical Study of Heart Failure with Left Ventricular Ejection Fraction Regimen Treated with Entresto" was retracted in 2023. Reasons: signs of a paper mill; suspected computer-generated content; unreliable results or conclusions; concerns about the data.

Serum NE reflecting the body's sympathetic nerve activity has been clinically confirmed to be associated with the regulation of cardiac function. When heart failure occurs, the cardiac compensatory mechanism rapidly activates the sympathetic nervous system, prompting the body to release a large amount of NE, resulting in an increase in the level of NE in the plasma. The continuous increase in NE will aggravate the hemodynamic disorder and increase the cardiac load and energy consumption, which promote myocardial cell apoptosis and necrosis. Therefore, the increase in serum NE level suggests the activation of sympathetic nerve and impaired myocardial function [22, 23]. Elevated serum AngII level will activate the sympathetic vasoconstrictor center and increase the vascular load and myocardial oxygen consumption. Elevated serum ALD levels can induce water and sodium retention and increase circulating blood volume, which aggravates myocardial injury and cardiomyocyte apoptosis. The elevated levels of MMP-9 often indicate decreased left ventricular function, myocardial remodeling, and myocardial damage. Therefore, the levels of NE, AngII, ALD, and MMP-9 in the two groups were decreased after treatment with a lower level in the treatment group, suggesting that Entresto exerted a certain myocardial protection effect through inhibition of the sympathetic nerve and the reduction of myocardial damage.

## 5. Conclusion

This study also examined whether Entresto clinically benefits patients with HFpEF. A prospective randomized controlled trial design was adopted, and a total of 78 patients with HFpEF were enrolled. Thirty-nine patients were treated with Entresto based on conventional treatment. The results showed that Entresto significantly reduced BNP level and clinical endpoint events. The left ventricular diastolic function index of the cardiogram, the 6-minute walk test, and the MLHFQ score was also significantly improved, and the therapeutic effect was significant without increasing the incidence of adverse reactions. The results of the present study suggest that Entresto can significantly improve the left ventricular diastolic function of patients with heart failure whose left ventricular ejection fraction is preserved with NYHA cardiac function classification of II ∼ III and improves patient quality of life. Therefore, Entresto is safe and effective, and worthy of clinical application. A larger-scale clinical trial, PARAGON (NCT01920711), has been launched for this patient population. The trial will enroll ∼4300 patients with LVEF >45% [24]. Whether Entresto can improve the prognosis of large-scale HFpEF patients is an important next step in evaluating the clinical effects of treatment [25, 26].

## Figures and Tables

**Table 1:** Comparison of echocardiographic indexes of two groups of patients before and after treatment.

Variables	Time	Control group	Entresto group
LVMI (g/m^2^)	Pre-treatment	139.85 ± 44.53	140.51 ± 45.25
	Posttreatment	112.55 ± 23.33^#^	105.37 ± 21.47^#*∗*^

LVEF (%)	Pre-treatment	52.14 ± 8.81	51.32 ± 8.74
	Posttreatment	54.33 ± 9.27^#^	57.58 ± 10.25^#*∗*^

LVEDD (mm)	Pre-treatment	49.5 ± 5.7	48.7 ± 5.6
	Posttreatment	47.6 ± 5.1	43.4 ± 4.8^#*∗*^

LVESD (mm)	Pre-treatment	36.8 ± 4.0	37.7 ± 4.2
	Posttreatment	35.0 ± 3.9^#^	31.3 ± 3.9^#*∗*^

E/E′ ratio	Pre-treatment	14.95 ± 3.82	15.12 ± 3.68
	Posttreatment	10.63 ± 2.14^#^	8.32 ± 1.66^#*∗*^

E/A ratio	Pre-treatment	0.76 ± 0.12	0.75 ± 0.12
	Posttreatment	0.82 ± 0.14	0.98 ± 0.15^#*∗*^

DT (ms)	Pre-treatment	285.52 ± 50.38	295.30 ± 55.74
	Posttreatment	254.85 ± 47.77^#^	233.65 ± 48.69^#*∗*^

Compared with before treatment ^#^*P* < 0.05, compared with the control group, ^*∗*^*P* < 0.05.

The article "Clinical Study of Heart Failure with Left Ventricular Ejection Fraction Regimen Treated with Entresto" was retracted in 2023. Reasons: signs of a paper mill; suspected computer-generated content; unreliable results or conclusions; concerns about the data.

**Table 2:** Comparison of plasma BNP levels of the two groups of patients before and after treatment.

Variable	Time	Control group	Entresto group
BNP (pg/ml)	Pre-treatment	631.6 ± 60.5	626.7 ± 57.8
	Posttreatment	566.4 ± 43.7	331.6 ± 40.6^#*∗*^

Compared with before treatment ^#^*P* < 0.05, compared with the control group, ^*∗*^*P* < 0.05.

**Table 3:** Comparison of 6MWD and quality of life between the two groups before and after treatment.

Variables	Time	Control group	Entresto group
6MWD	Pre-treatment	345.28 ± 32.72	340.82 ± 31.49
	Posttreatment	382.14 ± 45.51^#^	410.32 ± 52.50^#*∗*^

MLHFQ scores	Pre-treatment	68.39 ± 12.14	66.75 ± 11.53
	Posttreatment	44.20 ± 8.25^#^	38.32 ± 8.36^#*∗*^

Compared with before treatment ^#^*P* < 0.05, compared with the control group. ^*∗*^*P* < 0.05.

**Table 4:** Comparison of serum factor levels between the two groups before and after treatment.

Variables	Time	Control	Entresto group
NE (pmol/L)	Pre-treatment	2397.92 ± 370.28	2398.71 ± 369.57
	Posttreatment	1975.84 ± 293.42^#^	1702.96 ± 233.68^#*∗*^

AngII (ng/L)	Pre-treatment	134.78 ± 19.06	134.25 ± 18.94
	Posttreatment	119.49 ± 16.34^#^	108.32 ± 15.18^#*∗*^

ALD (pg/ml)	Pre-treatment	349.21 ± 83.52	348.95 ± 83.46
	Posttreatment	319.85 ± 74.61^#^	300.26 ± 65.23^#*∗*^

MMP-9 (*μ*g/L)	Pre-treatment	171.04 ± 27.13	170.89 ± 26.72
	Posttreatment	161.58 ± 20.37^#^	152.43 ± 18.65^#*∗*^

Compared with before treatment ^#^*P* < 0.05, compared with the control group, ^*∗*^*P* < 0.05.

**Table 5:** Comparison of the curative effect on cardiac function.

Group	*n*	Significantly effective (*n*, %)	Effective (*n*, %)	Ineffective (*n*, %)	Efficient (%)
Control	39	9 (23.08)	21 (53.85)	9 (23.08)	76.92
Entresto	39	17 (43.59)	20 (51.28)	2 (5.13)	94.87
*χ * ^2^					5.192
*P*					0.027

**Table 6:** Comparison of composite clinical endpoints between two groups of patients.

Group	*n*	*Endpoints*		*Adverse reactions*				
		Cardiovascular events	Worsening heart failure	Dizziness	Impaired kidney function	Hyperkalemia	Hypotension	Total
Control	39	7 (17.95)	6 (15.38)	3 (7.69)	1 (2.56)	0 (0.00)	1 (2.56)	5 (12.81)
Entresto	39	2 (5.13)	1 (2.56)	1 (2.56)	1 (2.56)	1 (2.56)	1 (2.56)	4 (10.24)
*χ * ^2^		7.562	6.654					2.562
*P*		0.013	0.025					0.078

## Data Availability

The simulation experiment data used to support the findings of this study are available from the corresponding author upon request.
